The article "Mechanism of Undergraduate Students' Waste Separation Behavior in the Environmentally Friendly Higher Education Mega Center of Guangzhou" was published in 2022. Journal: J Environ Public Health.

# Mechanism of Undergraduate Students' Waste Separation Behavior in the Environmentally Friendly Higher Education Mega Center of Guangzhou

**DOI:** 10.1155/2022/4475245

**Published:** 2022-07-30

**Authors:** Dong Wang, Weishan Chen, Xiarou Zheng, Yuxin Li

**Affiliations:** ^1^School of Management, Guangzhou University, Guangzhou 510006, China; ^2^School of Management, Shenzhen University, Shenzhen 518060, China

## Abstract

The volume of waste produced by aspects of both industrial life and daily life has increased in the past few years in conjunction with the rapidly growing economy in China. In urban areas, citizens consume more resources and produce much waste, which pollutes the environment. Many cities have proposed numerous regulations for waste separation to help build environmentally friendly cities. Plenty of studies tried to reveal the mechanism of residents' waste separation behavior in different theoretical perspectives but were unable to clarify the effect of waste separation factors in university. Moreover, the response and performance of undergraduate students after the waste separation regulations are proposed and are not well discussed. To clarify the mechanism of waste separation behavior in campus and evaluate the response and performance, in this study, a questionnaire is used to sample undergraduate students from the Higher Education Mega Center in Guangzhou. With the use of SPSS 23.0, this study conducts an empirical analysis; the results of which show that (1) environmental awareness and personal responsibility have a significant positive impact on behavior attitude; (2) convenience and economic cost have a significant positive impact on perceived behavior control; (3) intention has a partial mediating role between behavior attitude, subjective norms, and perceived behavior control; and (4) habits directly affect behavior and regulate the relationship between intention and behavior. The results will provide some meaningful implications for the government.

## 1. Introduction

China's urbanization process continues to develop; approximately 60.60% of the country's population was urbanized in 2019. At the same time, the rapid development of industrialization has resulted in a large consumption of resources, which results in a large volume of waste in urban cities being increasingly produced [1]. The waste in urban cities is officially called municipal solid waste (MSW), which is produced from aspects of residents' daily lives, public places, commercial departments, and public institutes [2]. As the largest waste producer in the world, China maintains an annual growth rate of 8%–10%, and many cities lack land resources for landfills [3], which indicates that landfills and incineration, as the main means of urban solid waste treatment in China, cannot keep up with the growth rate of waste generation. To build an environmentally friendly society in China, the government has proposed separation and evaluation standards for MSW since 2004, as well as building waste separation infrastructures. However, because of the lack of specific details on MSW separation, urban residents have little knowledge of MSW separation operations, and recycling MSW does not work well, which hurts the environment in urban districts.

The efficiency of MSW recycling and waste separation instruction is still not high in China. Eight Chinese cities, including Beijing and Shanghai, have begun to conduct MSW separation since 2000, but none of these cities have achieved the expected results [1]. In February 2019, the Ministry of Housing and Urban-Rural Development in China ordered all cities at the prefecture level and above to promote the separation of MSW. With the increase in various intelligent waste separation facilities in the streets, the arrangement of separation transport vehicles, and the promotion of volunteer community publicity, all aspects and links of these cities have begun to prepare for multifarious waste separation. However, the reality is not optimistic. According to the results of a public opinion survey conducted in Chongqing in April, more than 40% of respondents still feel that waste separation is problematic and difficult to operate [3].

The management of MSW is usually viewed as an important index of city governance. As a country with a large volume of waste production, the management of MSW is still weak in China. MSW is the main source of pollution for the urban environment, as well as an important aspect of the recycling perspective. Issues related to viewing MSW as a type of treasure and the recycling of these resources, including increasing their harmlessness and the overall amount of MSW, are becoming increasingly significant. The initial step of recycling MSW is waste separation from residents. Hence, there are a large number of studies focusing on revealing the mechanism of residents' waste separation behavior in different theoretical perspectives, with the aim to provide all residents and management departments with suitable waste separation instructions to followed by referenece [4–8]. However, most studies are sampled to the city residents. The undergraduate students who are well-educated will have positive passion in waste separation promotion in society. The effect of waste separation factors in university needs to be clarified. In addition, although there are abundant researches on the recycling of MSW from the social and psychological perspectives, the evaluation of the response and performance after the residents received the waste separation instruction is not well interpreted. Researchers have focused on the effecting factors and management of MSW separation behavior, and this information contributes to environmental protection regulation and environmentally friendly city building. These previous studies are common in proposing research models based on behavior theory; the main influencing factors in MSW separation behavior include but are not limited to low environmental protection intention, MSW separation instructions being difficult to follow, insufficient laws and regulations, little investment in MSW separation education, and a low level of infrastructure building. Further, the response and performance of the residents when they encountered these complex and difficult instructions are hard to evaluate. We thus propose the second research questions of this study as follows.

1. What are the influencing factors of waste separation behavior in undergraduate students and what are the effects among these identified influencing factors?
2. What is the response and performance of undergraduate students when faced with waste separation instructions?

To answer these questions, this study first proposes an instructive policy model of waste separation behavior and highlights the interaction of the influencing factors in the proposed research model, which contributes to the findings of previous studies in the model setting. Compared with the existing research model, behavior habits are taken to verify the moderating effect between behavior intention and waste separation behavior, and behavior intention is viewed as a mediating variable between attitude, subjective norms, and behavior control with regard to waste separation behavior. In the data sampling process, we collect information from undergraduate students in the Higher Education Mega Center in Guangzhou, which has a good waste separation area in an environmentally friendly city building. The results will provide some meaningful implications for the government. The second contribution of this study is revealing the waste separation mechanism in response to the incentive policy outlined by government. Via its research design, this study explores the interaction of all influencing factors based on the “execution-pull” mode, which underlies the effect mechanism under the incentive of government waste separation regulations. All the hypotheses are proposed and tested within the background of such pulling regulations, and the results are analyzed for ease of resident execution. Furthermore, the implications are discussed both theoretically and practically. Moreover, the variable measurements are based on combinations of previous studies and have higher reliability and validity after revision, which helps to provide new measurements for the empirical study of waste separation behavior.

This study is organized as follows. We review the literature in Section 2 to clearly define the connotation of waste separation behavior. In Section 3, based on the literature analysis of behavior theory, the hypotheses and research models are proposed. Then, the data and sampling are described in Section 4. The results are analyzed in Section 5. The discussion and conclusions are presented in Section 6. This study can improve the initiative of college students to participate in waste separation and the level of waste separation in China.

## 2. Literature Review

### 2.1. Waste Separation Behavior

Waste separation behavior is a specialized and specific environmental behavior. When defining its dimensions, we can refer to relevant studies on environmental behavior structure. In the field of social marketing, there are two main interpretations of environmental behavior; one interpretation focuses on the subject of the actor, agrees with the view that environmental choice behavior is actively chosen by the actor, and calls engaging in environmental behavior an “active choice,” while the other interpretation emphasizes external social structure, which restricts and influences environmental selection behavior and calls such behavior “passive selection” [9]. It can be seen that waste separation is “a complex process” [10, 11]. Foreign scholars began to pay attention to waste separation and recycling earlier; thus, their research level is higher. Wertz's research was first involved in the field of residential waste separation [12]. Based on the research results of Jenkins and Jarvinen, the influence of incentive and punishment measures on the waste separation participation rate has been verified [13]. Subsequently, in terms of policy factors, government financial input, knowledge publicity, and education have been suggested to have a direct or indirect impact on waste separation behavior.

The research of domestic scholars in this field is divided into the macro-policy environment level and micro-individual level. At the macro-level, scholars have analyzed the influence of social and economic levels, government assessment, laws and regulations, living habits, and other factors on residents' separation behavior. At the micro-level, Vu et al. proposed factors such as moral constraints, environmental awareness, environmental behavior and attitude, and environmental value from the internal perspective of residents [14]. Li et al. believed that the internal behavior and attitude of residents, such as responsibilities and obligations, under the coercion and stimulation of external factors, would play an important role in the efficiency of waste separation [15]. In the empirical field of large samples, Razali et al. took the waste separation policy of Guangzhou as a case study and found that from the perspective of policy marketing, various publicity channels, such as TV, newspaper, Internet, and face-to-face and government official channels, can increase the explanatory power of waste separation [4].

Previous studies have elaborated on various influencing factors of MSW separation at the macro- and micro-levels. However, more studies at the micro-level focus on testing behavioral intention, thereby ignoring the fact that one's willingness and actual behavior are not equivalent. In addition, although the advanced analytical framework and ideas of foreign research are of great significance to promote the theory and practice of waste recycling and utilization in China, the research conclusions and suggestions still need to be localized.

### 2.2. Factors Influencing Waste Separation Behavior

At present, waste classification factors are divided into psychological-level factors, situational-level factors, interaction factors, individual characteristics, etc.

Psychological-level factors include value factors, environmental cognition, adjustment focus, comfort preference, utility perception, and others. In terms of values factors, in a sample of British urban residents, Li et al. found that while social altruistic values are the main influence of a low-carbon lifestyle and ecological values are also a factor, care for the environment is not a main motivation, and changing one's original lifestyle is more due to the influence of human interests; therefore, the authors support the connection between altruistic values and low-carbon behavior [5]. In his research of low-carbon consumption behavior, Ajzen showed that such values are divided into conspicuous consumption values, emotional consumption values, economic consumption values, functional consumption values, and social consumption values [16].

In terms of environmental cognition, Zeng et al. argued that all human behaviors are related to factors such as cognition and emotion [6]. Wang et al. found that cognition can not only influence behavioral decisions at the conscious level but also work at the unconscious level, which can influence individual behavior through mechanisms such as habits [17]. In the field of environmental research, most scholars also agree with the view that cognition determines behavior. Environmental cognition refers to the individual's knowledge of environmental problems [18], recognition [19], concerns [20, 21], etc.

In terms of regulatory focus, behavior is an individual's psychological reaction to original cognitive factors, situational factors, the group atmosphere, and other information sources after processing feedback explicit activity. Included in an individual's processing of information sources is a process of regulation, and different attention tendencies will prompt him or her to choose different behavior strategies; thus, these tendencies can be used to adjust his or her focus for expression. Regulatory focusing is the specific psychological tendency of individuals to differently select and respond to external stimuli through self-regulation in cognition and decision-making processes, including promoting focusing and preventing focusing. In traditional motivation theory, the pleasure principle (Hedonic principle) of “seeking benefits and avoiding harm” is the dominant idea [22–25]. In terms of comfort preference factors, residents' participation in decisions related to environmental behaviors such as resource recovery also depends on their pursuit of comfort in many cases. In a survey of general environmental behaviors conducted among 2167 and 1250 residents in the Netherlands regarding household energy use behaviors, Wood and Neal [26] found that different types of environmental behaviors also have different mainly affected variables. When people engage in some environmental behavior that is not expensive and does not take much effort, ordinary attitude variables have a greater impact on behavior. De Bruijn et al. [27] used the comparative dynamic analysis method to analyze consumers' green ecological housing preferences. The results showed that environmental comfort parameters are one of the important influencing factors of green ecological demand.

Planning behavior theory states that the more resources and opportunities a person senses when performing a particular behavior, the fewer anticipated barriers are likely to occur, the stronger the perceived behavioral control will be, and the more the corresponding behavior is likely to occur. In terms of utility perception, Lu et al. [28] found that reducing the behavioral costs to individuals can contribute to residents' recycling behavior. That is, in addition to the convenience and ease of use with regard to comfort characteristics, the “benefits” or utility perceived by individuals will often determine whether they will classify the waste. Miafodzyeva and Brandt [29] pointed out that college students with more awareness of waste pollution and waste harm are more aware of the significance of waste source classification and are thus more willing to participate in waste classification activities. Based on this, this study will further explore the mechanism of urban residents' utility perception in various aspects on their waste classification behavior.

Scenario-level factors include policy factors, product and facility factors, and group specification factors. Diekmann and Preisendörfer [30] divided the influencing factors of situational factors on urban residents' energy-saving behavior into policy class elements and product factors, including policy factors such as policy implementation and validity, mainly through economic policies and policy guides; the authors used residents to measure the implementation of energy-saving policy strength and validity. Glick et al. [31] summarized the situational factors affecting the low-carbon consumption behavior of urban residents into six aspects, namely policies and regulations, social norms, publicity and education, and technology maturity. Rajapaksa et al. [32] divided the environmental behavior of urban residents into three aspects, namely behavior constraints, public norms, and reward and punishment mechanisms, among which behavior constraints are mainly reflected through government policies. Based on this, this study believes that the popularity of waste classification behavior control policies will affect the implementation of waste classification behavior.

In terms of product and facility factors, Masud et al. [33] found that although people pay more attention to environmental issues and hold positive environmental values, their environmental behaviors are also affected by the local situation and atmosphere. If green products are not widely available geographically, residents will still choose more environmentally friendly procurement behaviors. Liu et al. [34] also pointed out that the government's partial provision of convenient sorting facilities and collection services will promote active public participation in the source sorting of food waste. It can be seen that the maturity and popularization of classified recycling technologies, products, and classification facilities will directly affect the convenience level of individuals with regard to engaging in waste classification, reduce the cost of individual time and energy, and help promote residents form habits related to waste classification.

In terms of group specification factors, Wang et al. showed that if one's friends actively participate in waste classification, then an individual is more willing to make an effort to participate in waste field-level classification [35]. Bueno and Valente [36], using both planning behavior theory and a questionnaire analysis of Chinese Guangdong residents, found that an individual's attitude, subjective norms, perceptual behavior control, intention, and situation can significantly predict family waste classification behavior; the authors also pointed out that moral obligation-oriented propaganda and advocacy aiming to improve the participation rate of the prefecture-level classification are particularly effective.

Individual statistical characteristics have long been considered by scholars to have important effects on the behavior of individuals. Dean et al. [37] argued that demographic characteristics, such as education background, social status, and income, can not only reflect people's cognition of environmental problems and their ability to solve environmental problems but also even predict their environmental behavior to a certain extent. In the study of environmental protection behaviors such as waste classification, many scholars have obtained interesting conclusions. Bagozzi et al. [38] found that women are more involved in environmental behaviors such as waste management than men. An analysis of typical sociodemographic data from recyclers by Mak et al. [39] suggested that well-educated, affluent elderly residents are more likely to participate in waste separation. However, Mak et al. [39] also found different conclusions; e.g., they pointed out that low-income residents are positively associated with environmental behavior. Lu et al. [28] studied the source classification activities of residential organic waste through observation experiments and found that the housing style of residents affects the amount of household waste production and that families with smaller residential areas have higher efficiency in source classification than those with larger residential areas. Hafner et al. [40] pointed out that the factors affecting residents' participation in recycling include not only recycling awareness and motivation but also household characteristics, some of which can have a large impact on such behavior; i.e., larger households have higher levels of recycling willingness and participation rates than smaller households. Masud et al. [33] also noted that demographic factors such as age, gender, and education can influence waste management behavior.

In addition, Wang et al. pointed out that the interpersonal behavior model is most closely related to low-carbon consumption behavior because low-carbon consumption is a daily trivial behavior consisting of habits and regularity [35]. Therefore, it can be considered that the model has profound reference significance for the study of low-carbon consumption behavior [27, 41, 42]. For example, Jager [43] used interpersonal relationship theory as a critical framework to explore its effect on Thai families' participation in recycling behavior from the perspective of habits. The results show that recycling willingness, recycling habits, recycling ability, facility conditions, and the adequacy of recycling information have significant predictive effects on recycling behavior. The study also found that the higher the degree of habit is, the less dependent the recycling behavior is on intention [28, 29, 43].

### 2.3. Mechanism of Waste Separation Behavior

Based on this theory, Bargh et al. [42] set up an integrated MSW management model and found that recycling behavior is largely determined by behavioral intention and behavior control. In addition, behavioral intention is affected by attitude, social norms, and behavior control. This conclusion reflects the reasonability of the theory of planned behavior used to explain and forecast the recycling behavior of MSW separation. Based on the theory of planned behavior, Wang et al. [35] used data from a questionnaire survey to analyze the influencing factors of public participation in the source classification of food waste. The results indicated that under the condition that local authorities fully prepared the opportunities, facilities, and knowledge related to the source classification of waste, the public had a high level of willingness to participate in the source classification of waste. Moreover, good moral values and situational factors, such as stockpiling convenience and collection time, can also increase public participation in waste separation. Saba et al. [24] applied the rebound effect to the study of environmental policy and considered the rebound effect to be an individual behavior or a response of the system to policies aiming to mitigate environmental impacts, which will counteract the policy and the utility of technology. Because of this derivative reaction, some ecological policies are not only less effective than expected but also have a negative impact. Usui and Takeuchi [44] used the connotation of the rebound effect to explain the change in MSW reduction through 8 years of tracing investigation in their study.

Liu et al. [34] reviewed and summarized the municipal solid waste control policies of some industrially developed countries (including Europe, Japan, and the USA) and argued that these countries have generally formulated three types of waste control policies, namely law, economy, and management policies. Kang et al. [45] divided the Chinese municipal solid waste regulation policy into three categories, namely the downstream policy, the upstream policy, and the comprehensive policy; the downstream policy is directly related to domestic waste disposal and consumption behavior, the upstream policy is related to manufacturers' production behavior, and the comprehensive policy includes policies that affect both manufacturers and urban residents. Wu et al. [46] argued that the regulation and control policies for municipal solid waste issued by Chinese governments at all levels basically cover three main regulatory means, namely value-added tax collection and backwardation, the household waste charging system, and recycling subsidy policy. From the perspective of regulators, Fu et al. [7] summarized Japan's waste control policies into four categories, namely civic participation, education and publicity, legal constraints, and government incentives. In behavior-related research theory, cognition is the basis of behavior willingness; the cognition of urban residents is reflected in the degree of understanding and recognition of the policy content, while behavior willingness is reflected in the degree of policy compliance and publicizing the policy to others, thus encouraging more people to follow. In their study on the new rural insurance subsidy policies, Wu et al. [47] showed that policy cognition can influence individuals' behavioral choice. However, some scholars believe that there is no inevitable connection between individual policy cognition and behavior choice; for example, in regard to the public attitude toward mandatory water-saving policy and the policy effect of public cognition, research has found that even if the local residents do not support the mandatory water-saving policy, the policy will still be effective, and residents will reduce their water usage.

## 3. Hypothesis and Models

### 3.1. Research Hypothesis

#### 3.1.1. Influence of Behavioral Attitude on Waste Separation Behavior

Behavioral attitude is generally defined by scholars as the psychological tendency to like something.

In the research of social marketing, behavior and attitude have undoubtedly become internal factors of individuals. Most studies show that an individual's specific behavior and attitude related to the environment can affect his or her environmental behavior. Based on previous literature, Lu et al. proposed that in the research field of green purchasing behavior, behavioral attitude has the greatest predictive power for purchasing behavior [28]. Miafodzyeva et al. used the probit model as a tool to study the intention and behavior of waste separation of residents and found that residents with higher environmental attitudes are more likely to have the intention of engaging in waste separation [29].

#### 3.1.2. The Influence of Subjective Norms on the Waste Separation Behavior

Subjective norms mean that individual behavior decisions are influenced by both others and society [30–32]. Some scholars have proposed that in different cultural backgrounds, the social relations around individuals will either promote or restrict individuals' behavioral decisions to varying degrees [48].

In China, people often depend on the attitudes of those around them to decide to do something or engage in a certain behavior. This shows that subjective norms emphasize the role of social influence in waste separation. Different social groups, such as family members and neighbors, influence individual decisions. Social dilemmas may arise when individuals change their actions to address environmental problems. Thus, one hopes to conform to the opinions of others and integrate into one's community by engaging in support for environmental protection. Therefore, subjective norms affect individuals' thinking and decision-making regarding the implementation of a certain behavior [33].

In the field of environmental behavior research, Liu et al. took residents as the research objects and pointed out that subjective norms have a significant positive impact on residents' intention of engaging in waste separation [34]. Wang et al. studied the transformation from attitude to behavior of urban residents in waste separation, concretized the subjective normative definition, and argued that residents with strong collectivist values in China's special national conditions are more inclined to support waste separation [35]. Therefore, to clarify the working principle of subjective norms, this study will also discuss the intention and internal mechanism of subjective norms on waste separation behavior.

#### 3.1.3. The Influence of Perceptual Behavioral Control on the Separation Behavior

Perceptual behavioral control is defined as an individual's self-perception and judgment of a certain behavior [36, 40, 49]. As one of a large number of studies based on TPB theory, Lu et al. studied the influencing factors of consumers' behavioral intention of e-waste investment and payment in Henan Province, where economic development is relatively slow; the authors showed that perceptual behavioral control has a significant impact on the behavioral intention of e-waste investment and payment [28]. Fan et al. studied the recycling behavior of waste household appliances and electronic products and found that past recycling habits and perceptual behavioral control are significant factors affecting recycling behavior [50]. Dean et al. took residents as the research object and found that reducing the implementation difficulty of waste separation could more easily enhance residents' perceptual behavioral control and thus trigger waste separation behavior [37].

In daily behaviors, such as high-frequency waste separation, although individuals are more dependent on habits to decide whether to implement waste separation, the convenience of separation facilities will still affect individuals' perception of the difficulty of the behavior, which will thus influence the participation rate of waste separation behavior.

#### 3.1.4. Influence of Behavioral Intention

Intention refers to the stabilization of an individual psychological state, which forms a behavioral motivation, which in turn directly affects behavior. In a large number of empirical studies in the field of social marketing, scholars have found that for simple waste separation, behavioral intention not only is affected by behavioral attitude, subjective norms, and other factors but also directly and significantly predicts recycling behavior. Bagozzi et al. used the goal-directed behavior (MGB) model to predict the intention to use public transportation instead of private cars to travel to work; furthermore, research on recycling household waste has tested a similar hypothesis and has pointed out the predictive role of behavioral attitude, subjective norms, and perceptual control in pro-environmental behavioral intention [38].

In this study, behavioral intention and behavior are distinguished, and the relationship between these factors and related rational factors, such as behavioral attitude, subjective norms, and perceived behavioral control, is explored.

Based on the above analysis, we propose the following hypotheses:

  H1: the behavioral attitude of college students toward waste separation behavior has a significant positive impact on waste separation behavior.
  H2: the subjective norms of the waste separation behavior of college students have a significant positive impact on waste separation behavior.
  H3: the PBC of college students has a significant positive impact on waste separation behavior.
  H4: the behavioral intention of engaging in waste separation behavior plays a mediating role in the behavior attitude and waste separation behavior of college students.
  H5: the behavioral intention of college students regarding waste separation behavior plays an intermediary role in subjective norms and waste separation behavior.
  H6: the behavioral intention of engaging in waste separation behavior plays a mediating role in the perceived behavioral control and waste separation behavior of college students.

#### 3.1.5. The Moderating Effect of Irrational Factor Habits

As mentioned above, other scholars have found in their studies that there is a lack of necessary transformational element between intention and behavior, which plays a mediating or moderating role between them [39, 51–53]. Some scholars have verified that habits have a direct effect on behaviors and that habits and behavioral intentions jointly affect behaviors. In addition, Best and Kneip found in his study on the choice of driving mode of 1000 drivers that drivers with strong car habits have a weaker intention to use public transport, while drivers with weak car habits have a stronger intention to use public transport. In other words, car driving habits are expected to moderate the intention-behavior relationship of public transport use; that is, habits have a moderating effect in the medium term of the intention-behavior relationship [54]. Therefore, based on the theory of interpersonal behavior and other related studies, this study will establish a model with which to study the irrational factors of the relationship between habits and behavioral intentions, as well as the influence of behaviors.

Based on the above analysis, this study proposes the following hypothesis:

  H7: waste separation habits of college students play a moderating role in the relationship between behavioral intention and waste separation behavior.

#### 3.1.6. Influencing Factors of Behavior and Attitude

Environmental awareness refers to behavior in which individuals choose to participate in environmental protection based on their values of environmental protection after understanding and paying attention to environmental protection conditions, which is eventually reflected in their environmental protection behavior [55–57]. Chan et al. used the linear structural equation method to explore the difference in family participation rates in recycling programs implemented by urban and suburban communities and found that environmental awareness has a significant impact on individual recycling behavior and attitude [58]. Bamberg argued that general behavioral attitudes cannot directly affect specific environmental behaviors and that only the specific situational cognition of significant consequences associated with specific behaviors can be the direct determinant of specific behaviors. General behavior attitude is an important indirect factor influencing specific behavior. That is, environmental awareness needs to be internalized into behavioral attitudes and subjective norms to indirectly influence specific environmental behaviors [19]. Based on this, the following hypothesis is proposed in this study:

  H8: the environmental awareness of college students has a significant positive impact on their behavior and attitude.

Personal responsibility is one of the important psychological variables affecting individual environmental behavior. This factor refers to the individual's moral cognition and sense of mission about carrying out certain environmental behavior. On the whole, the existing studies all agree that sense of responsibility is one of the factors affecting residents' environmental behavior. Disagreement exists only regarding whether the influence path is direct, indirect, or both. Ghani et al. studied the influence mechanism of green consumption on internal psychological factors and external policy intervention variables of Chinese consumers, investigated the indirect path of responsibility on behavior, and pointed out that individual responsibility has a positive effect on the behavior and attitude of waste disposal [59].

In particular, individuals with a higher sense of responsibility are more concerned about environmental protection, regard such protection as a moral constraint and advocacy principle, and are more likely to respond to environmental policies and actively participate in environmental protection behaviors. In contrast, individuals with a lower sense of responsibility are more likely to ignore environmental problems and remain indifferent to the management of waste separation behavior.

Based on the abovementioned information, this study also adopts the indirect path and puts forward the following hypothesis:

  H9: college students' sense of personal responsibility has a significant positive impact on their behavior and attitude.

#### 3.1.7. Influencing Factors of Perceptual Behavioral Control

As mentioned above, convenience and economic cost are taken as antecedent variables of perceived behavior control in this study. Hebrok et al. found in discussing the influence mechanism of perceived behavioral control on sustainable consumption behavior that convenience affects control belief and thus perceptual behavioral control [60]. In practice, individuals are more likely to properly dispose of waste due to the proximity of waste collection facilities and the low cost of consumption. When waste collection behavior is difficult to implement, individuals are more willing to choose to dispose of waste at will.

Based on this, the following hypothesis is proposed in this study:

  H10: the convenience of waste separation behavior has a significant positive influence on the perceived behavior control of college students.

In this study, economic cost is defined as the economic cost paid by college students in waste separation. Leeabai et al. [61] pointed out that recycling is seen as expensive among residents because it requires time and effort to store, sort, and transport recyclable materials to recycling facilities. In Nilashi et al. [62] research on the ranking of psychological factors that influence managers' adoption of green, economic cost-benefit assessment analyzed the dimensions of perceived behavioral control; it was concluded that economic cost-benefit assessment occupies fourth place in the ranking list of influencing factors [60].

In reality, a high economic cost increases the difficulty of implementing an actual behavior, increases the obstacles for consumers to perform a classified behavior, and thus reduces the perceived behavioral control of consumers. In this study, economic cost was innovatively added into the model as an antecedent variable of perceived behavior control.

Based on this, the following hypothesis is proposed in this study:

  H11: the economic cost of waste separation has a significant negative influence on the perceived behavior control of college students.

### 3.2. Research Model

Through literature analysis, this study ultimately builds an influencing mechanism model of the waste separation behavior of college students (Figure 1). From the perspective of consumers, there are two main factors that affect waste separation behavior, namely rational factors, including behavior attitude, subjective norms and perceptual behavioral control, and irrational factors, including habits. In addition, “environmental awareness” and “personal responsibility” were taken as antecedent variables of “behavior attitude.” On the other hand, convenience and economic cost were taken as antecedent variables of perceived behavioral control.

## 4. Data and Variables

### 4.1. Variables and Measurement

This study focuses on college students in the Higher Education Mega Center in Guangzhou. According to the maturity scale, the operational definition of each variable in this study is clarified, and a scale suitable for the context of this study is developed. The items are summarized in Table 1.

### 4.2. Data

#### 4.2.1. Sampling

This study selects college students from the Higher Education Mega Center in Guangzhou as the research object, including college students in various schools, grades, and majors. With the implementation of waste separation, universities located in the Higher Education Mega Center in Guangzhou have set up waste separation and recycling measures in many places on campus, especially to encourage students to classify kitchen waste, harmful waste, and recyclable waste in such accommodations. The topic and upsurge of waste separation have thus emerged, and various college students hold different opinions about and suggestions regarding waste separation behavior. Therefore, this study selects college students who are participating in and those who are not participating in waste separation in the Higher Education Mega Center in Guangzhou as research objects, which will be beneficial to obtaining more effective and accurate data.

In this study, five-point Likert-type subscales were used to measure variables, and accurate and undisputed statements were used to prompt respondents to answer questions. The questionnaire in this study mainly includes the following three parts.

The first part asks the subjects to provide their personal information, including gender, educational background, school type, major type, monthly income, and other basic information about the respondents. Considering that the above factors may have an impact on waste separation behavior, this study uses them as control variables.

In the second part, the respondents are asked to answer observation questions related to various variables according to their actual situation, including behavior attitude, subjective norms, perceived behavioral control, behavioral intentions, and habits of the respondents about waste separation behavior.

Behavioral attitude questions 1–3 used the following answer options: “1” means “strongly disagree,” “2” means “disagree,” “3” means “general,” “4” means “agree,” and “5” means “strongly agree.” Subjective norm questions 1–3 used an answer option range, where option “1” means “no effect” and “5” means “high degree of effect.” The perceptual behavioral control, intention, habit, behavior, and other variables used an answer option range, where “1” represents “strongly disagree” and “5” represents “disagree.”

The third part measures the convenience, economic cost, environmental awareness, and personal responsibility of waste separation. On the utilized answer scale, 1 indicates “strongly disagree” and 5 indicates “disagree.”

#### 4.2.2. Questionnaire

To improve the reliability and validity of the scale, questionnaires were distributed to the respondents in advance as a pretest questionnaire. The final formal questionnaire was determined according to the structure and framework of the questionnaire.

This study adopted the method of a self-report questionnaire, and the subjects were asked to complete the questionnaire in a self-report manner. The subjects were not disturbed or guided by any questions. To collect accurate and effective data, not only were the respondents strictly controlled, but necessary screening was also carried out on the collected questionnaires for hypothesis verification.

### 4.3. Pretest

#### 4.3.1. Pretest Descriptive Statistics

In the pretest, 165 questionnaires were sent out in the form of a network, and 158 were recovered, among which 149 valid questionnaires were obtained after 9 invalid questionnaires were deleted. The structure of the recovered samples is shown in Table 2.

#### 4.3.2. Pretest Reliability and Validity

The pretest questionnaire was designed to measure the reliability of the scale through reliability and validity analysis. If the following two criteria are met, the questionnaire has a certain degree of reliability:

1. Cronbach's *α* value is greater than 0.7.
2. After rotation with the maximum variance method, the absolute value of the factor load is greater than 0.5.

According to general statistics, Cronbach's alpha reliability coefficient of 0.60–0.65 is untrustworthy, a coefficient of 0.65–0.70 is the minimum acceptable value, a coefficient of 0.70–0.80 is fairly good, and a coefficient of 0.80–0.90 is good. According to the test results of this scale (in Table 3), Cronbach's alpha coefficients are all higher than 0.7, indicating that the scale is highly reliable. Since the coefficients of convenience and economic cost did not meet these standards, when the coefficients of convenience question 2 and economic cost question 3 were deleted, it was found that the increased coefficients now meet the standards. Therefore, we decided to delete convenience question 2 and economic cost question 3.

The KMO value is intended to test whether a variable is suitable for factor analysis. The questionnaire KMO value of this study was >0.6, and the Bartlett sphericity test also passed the significance test (in Table 4). Since both items met the criteria, the variables could be analyzed by factor analysis. After removing convenience question 2 and economic cost question 3 due to low-reliability levels, the value was more in line with the standard, which means that it was suitable for factor analysis.

## 5. Analysis

### 5.1. Descriptive Statistical Analysis of Samples

This questionnaire was officially distributed to college students in the Higher Education Mega Center in Guangzhou. A total of 436 questionnaires were ultimately collected in this study. After deleting invalid questionnaires with serious problems, 400 valid questionnaires were ultimately collected, with an effective recovery rate of 91.7% (in Table 5).

### 5.2. Reliability and Validity Analysis

#### 5.2.1. The Reliability Analysis

Reliability is intended to measure whether the questionnaire items have internal consistency. The threshold of Cronbach's *α* > 0.7 was used to test the reliability of the questionnaire.

As shown in Table 6, the coefficient of behavioral attitude, subjective norms, perceived behavioral control, habits, behavioral intention, convenience, economic cost, environmental awareness, personal responsibility, and Cronbach's *α* was 0.811, 0.805, 0.739, 0.880, 0.899, 0.983, 0.788, 0.713, 0.824, and 0.783, respectively. The data all met the requirements; thus, it can be seen that the internal consistency of the measurement scale in this study is good.

#### 5.2.2. Validity of the Test

KMO and Bartlett's tests are used to observe whether variables are suitable for factor analysis. The KMO value in this study was 0.780, which means that the KMO was greater than 0.7. The Bartlett sphericity test had a significance of 0.000, indicating that factor analysis could be performed (in Table 7).

Factor attribution can be determined according to the results (as shown in Table 8), among which 9 questions ranging from habit 1 to habit 9 were assigned to Factor 1. Three questions of behavioral attitude (1–3) were assigned to Factor 2; the three items ranging from subjective norm 1 to subjective norm 3 were assigned to Factor 3; the three questions of perceived behavioral control (1–3) were assigned to Factor 4; the two questions ranging from convenience 1 to convenience 2 were assigned to Factor 5; and the two questions ranging from behavioral intention 1 to behavioral intention 2 were assigned to Factor 6. The two items ranging from personal responsibility 1 to personal responsibility 2 were assigned to Factor 7; the two items ranging from economic cost 1 to economic cost 2 were assigned to Factor 8; the two questions ranging from behavior 1 to behavior 2 were assigned to Factor 9; and the two questions ranging from environmental awareness 1 to environmental awareness 2 were assigned to Factor 10. The factor loadings described above were all greater than 0.7. A total of 10 factors with eigenvalues greater than 1 were extracted, and their cumulative variance contribution rate was 72.290%, which is greater than 60%. Thus, it met the criterion of the factor loading being greater than 0.7, thereby indicating the good content validity of the scale. The component matrix after rotation is shown in Table 9.

### 5.3. Correlation Analysis

Correlation analysis measures the strength of linear relationships between variables. The Pearson coefficient indicates the significance of the strength of the relationship between variables. The closer the absolute value of the Pearson coefficient is to 1, the stronger the correlation between variables is. The correlation analysis results of this study are shown in Table 8.

### 5.4. Regression Analysis

Regression analysis aims to study the interdependent quantitative relationship between two or more variables and to judge the explanatory variables leading to the change in the dependent variables, as well as the magnitude and direction of such influence by the size of the regression coefficient and positive and negative signs. To be statistically significant, the regression coefficient also needs to be tested for significance according to the *t* value. In this study, regression analysis is used to test the statistical relationship between variables. The regression analysis results are shown in Tables 10 and 11.

#### 5.4.1. Regression Analysis of Environmental Awareness, Personal Responsibility, and Behavior Attitude

In Table 12, Model 1.1 takes behavioral attitude as the dependent variable; gender, educational background, type of school, type of major, and average monthly income as the control variables; and environmental awareness as the independent variable. From the adjusted *R*^2^, the regression equation can explain 8.0% of the total variation. The regression coefficient *β*-value of environmental awareness in the model is 0.235, and the *t* value passes the significance test; that is, environmental awareness has a positive effect on behavior and attitude. Thus, Hypothesis H8 is verified.

In Model 1.2, behavioral attitude was taken as the dependent variable; gender, educational background, school type, major type, and average monthly income were taken as the control variables; and personal responsibility was taken as the independent variable. From the adjusted *R*^2^, the regression equation can explain 8.1% of the total variation. The regression coefficient *β*-value of personal responsibility in the model is 0.237, and the *t* value passes the significance test; that is, personal responsibility has a positive effect on behavior and attitude. Thus, Hypothesis H9 is verified.

#### 5.4.2. Regression Analysis of Economic Cost, Convenience, and Perceived Behavioral Control

In Table 10, Model 2.1 took perceptual behavior control as the dependent variable; gender, educational background, school type, major type, and average monthly income as the control variables; and economic cost as the independent variable. From the adjusted *R*^2^, the regression equation explained 6.9% of the total variation. The regression coefficient *β*-value of economic cost in the model is −0.257, and the *t* value passes the significance test; that is, economic cost has a negative effect on perceived behavior control. Thus, Hypothesis H11 is verified.

Model 2.2 took perceived behavior control as the dependent variable; gender, educational background, school type, major type, and average monthly income as the control variables; and convenience as the independent variable. From adjusted *R*^2^, the regression equation explained 3.6% of the total variation. In the model, the regression coefficient *β*-value of convenience is 0.182, and the *t* value passes the significance test, indicating that convenience has a positive effect on perceived behavioral control. Thus, Hypothesis H10 is verified.

#### 5.4.3. Mediating Effect

According to the research model and hypotheses in this study and according to the commonly used testing methods of mediation effect models, the model was constructed in three steps for testing: (1) Model 3.1, where the regression effects of independent variables' behavior attitude, subjective norms, and perceived behavior control on the behavior of outcome variables; (2) Model 3.2, where the regression effect of independent variables' behavioral attitudes, subjective norms, and perceived behavioral control on the mediating variables' behavioral intentions; and (3) Model 3.3, where the regression effect of behavioral intention of the mediating variable on the behavior of outcome variables. Gender, educational background, type of school, type of major, and average monthly income were added to the model as control variables.

*(1). Analysis of the Mediating Effect of Behavioral Intention on Behavioral Attitude-Waste Separation Behavior*. The test results are shown in Table 11. The adjusted *R*^2^ increased from 0.048 to 0.123; that is, the explanatory power of the model for waste separation behavior increased by 7.5% after the inclusion of behavioral intention. Although the *β*-value of behavioral attitude decreased gradually from 0.183 (*t* = 3.676, *P* < 0.001) to 0.117 (*t* = 2.379, *P* < 0.05), it was still significant. This proves that behavioral intention plays a partially mediating role in the relationship between behavioral attitude and waste separation behavior. Thus, hypotheses H1 and H4 are both verified.

*(2) Analysis of the Mediating Effect of Behavioral Intention on Subjective Normal-Waste Separation Behavior*. The test results are shown in Table 13. The adjusted *R*^2^ increased from 0.043 to 0.121; that is, the explanatory power of the model for waste separation behavior increased by 7.8% after the inclusion of behavioral intention. Although the subjective norm *β*-value decreased gradually from 0.170 (*t* = 3.412, *P* < 0.01) to 0.107 (*t* = 2.196, *P* < 0.05), it was still significant. This proves that behavioral intention plays a partially mediating role in the relationship between behavioral attitude and waste separation behavior. Thus, hypotheses H2 and H5 are verified.

*(3). Analysis of the Mediating Effect of Behavioral Intention on Perceived Behavioral Control-Waste Separation Behavior*. The test results are shown in Table 14. The adjusted *R*^2^ increased from 0.044 to 0.120; that is, the explanatory power of the model for waste separation behavior increased by 7.6% after the inclusion of behavioral intention. Although the *β*-value of perceptual behavioral control decreased gradually from 0.170 (*t* = 3.452, *P* < 0.01) to 0.104 (*t* = 2.128, *P* < 0.05), it remained significant. It can be proven that behavioral intention plays a partially mediating role in the relationship between perceived behavioral control and waste separation behavior. Thus, hypotheses H3 and H6 are verified.

#### 5.4.4. Regulating Effect

In this study, the moderating variables of habits are tested by a regression analysis of the moderating effects. First, major type was taken as a control variable in Model 4.1. Then, a regression model of behavioral intention on behavior was constructed in Model 4.2. A regression model of the habit variable on behavior was added in Model 4.3, and a regression model of the moderating effect of the habit and intention interaction on behavior was added in Model 4.4. Gender, educational background, type of school, type of major, and average monthly income were added to the moderating effect analysis as control variables.

The data analysis results are shown in Table 15. According to the adjusted *R*^2^ of Model 4.2, the explanatory power of behavioral intention increased by 9.5%. The *F* value was 9.435 (*P* < 0.001), which was statistically significant. When habits were included, the explanatory power of behavioral intention reached 13.7%, and the *F* value was 10.034 (*P* < 0.001). Thus, Model 4.3 shows that habits have a significant positive effect on behaviors. Interaction terms were added in Model 4.4, and it can be seen from the adjusted *R*^2^ that the explanatory power reached 14.4%; also, considering the positive and negative values of interaction terms (*β* = −0.099; *t* = −2.067, *P* < 0.05), it can be seen that interaction terms have a significant negative impact on behavior prediction.

In conclusion, waste separation intention and habits can jointly predict waste separation behavior. Such habits play a negative regulating role in behavioral intention and behavior. College students who have the habit of daily waste separation are largely in an “unconscious” state when choosing environmental behaviors. They do not find that waste separation has been implemented until the completion of waste separation. However, for college students who do not have the habit of environmental protection, their choice of environmental behavior is largely based on rational consideration, and factors such as separation awareness and convenience are more likely to become important factors affecting their behavior intention and behavior. According to the analysis results, Hypothesis H7 is verified.

## 6. Conclusion and Discussion

### 6.1. Conclusion

According to the results of the analyses, the hypotheses proposed in this study have been verified accordingly, and the verification results are shown in Table 16.

This study is mainly divided into three parts. The first part discusses the influence of environmental awareness on attitude, the influence of personal responsibility on attitude, the influence of convenience on perceived behavioral control, and the influence of economic cost on perceived behavioral control. Hypotheses H8, H9, H10, and H11 are all shown to be valid. The second part focuses on college students' attitudes and waste separation behavior to determine whether there is an intermediary effect, on subjective norms and behavior to determine whether there is an intermediary effect, and on perceived behavior control and behavior to determine whether there is an intermediary effect; H1, H2, H3, H4, H5, and H6 are supported. The third part focuses on whether the waste separation habit of college students has a moderating effect on the impact of behavioral intention on waste separation behavior, which supports H7.

### 6.2. Discussion

#### 6.2.1. The Influence of Environmental Awareness and Personal Responsibility on Attitude

This study discusses the influence of environmental awareness and personal responsibility on attitude. It can be seen from the verification results that the environmental awareness of college students has a significant positive impact on their attitude; that is, when college students have environmental awareness, they are more enthusiastic about waste separation. This outcome is consistent with the results of domestic and foreign scholars in the study of waste separation behavior; that is, environmental awareness affects behavioral intention by affecting specific behavioral attitudes. Moreover, this study also found that college students' environmental awareness of waste separation has significant differences based on educational background. Lansana et al. [63] also concluded from an analysis of roadside waste recycling behavior in suburban communities that the education level and other variables of urban community residents affect their environmental awareness, evaluation of waste recycling operation policies, attention to the economy, and overall recycling behavior. Therefore, educational background causes differences in environmental awareness, which leads to making different choices for waste separation.

In addition, this study also proves that college students' sense of personal responsibility has a significant positive impact on their attitude; that is, when college students have a sense of personal responsibility, their enthusiasm to participate in waste separation is higher. This is consistent with the research results of domestic and foreign scholars on waste separation behavior; that is, personal responsibility affects behavioral intention by influencing specific behavioral attitudes. Moreover, this study also found that college students' personal responsibility for waste separation has significant differences in regard to educational background.

College students, as one of the groups often exposed to environmental protection education, understand the responsibility psychology and moral standards attached to the premise of recognizing environmental conditions and understanding environmental protection rules; thus, they have the cognition, belief, and value perception of classified behaviors, which means that they are more likely to have the consciousness to participate in environmental behaviors.

#### 6.2.2. The Effect of Convenience and Economic Cost on Perceived Behavior Control

This study discusses the influence of convenience on perceived behavior control and economic cost on perceived behavior control. From the verification results, it can be seen that the convenience of waste separation behavior has a significant positive impact on the perceived behavior control of college students; that is, recycling measures are more convenient for college students. For example, when the distance of recycling equipment is shorter and the separation rules are simpler, the participation rate of college students in waste separation behavior is higher. Few domestic and foreign social marketing studies take convenience as an antecedent variable of perceived behavior control to explore the internal relationship between the two. Through empirical research, this study found that convenience affects behavioral intention by influencing perceived behavioral control, which provides a new idea with which to enrich the research on perceived behavioral control of environmental behavior theory.

In addition, this study has also proven that the economic cost of waste separation has a negative impact on the perceived behavior control of college students; that is, when the economic cost of waste separation is lower or the economic return is higher, the participation rate of college students in waste separation behavior is higher. In most studies, economic cost is one of the situational factors affecting environmental behavior. This study innovatively takes economic cost as the antecedent variable of perceived behavior control to study the internal influence of both. The results show that economic cost affects behavioral intention by influencing perceived behavioral control, which can be used as a reference to clarify the complex mechanism of economic cost and perceived behavioral control on environmental behavior.

The convenience and economic cost of classifying behavior will affect the perceived difficulty of college students in classifying individual waste. When college students perceive classifying behavior more easily, their perceived hindrance factors will be reduced, which will thus increase the possibility of them participating in environmental behavior.

### 6.3. Implications

The research conclusions of this study can be applied to other similar behaviors with high frequency. The research conclusions can provide many useful references in theory and practice for the field of waste separation.

First, from a theoretical perspective, the results of verifying the influencing mechanism model of college students' waste separation behavior show that (1) Rational waste separation behavior intention can influence waste separation behavior, while rational behavior intention is affected by attitude, subjective norms, and perceptual behavioral control. (2) College students' waste separation behavior has a significant negative moderating effect on the relationship between behavioral intention and waste separation behavior. (3) Environmental awareness and personal responsibility have a significant positive impact on attitudes. Therefore, guidance strategies that aim to change the current situation can be proposed from the aspects of improving environmental awareness and personal responsibility. (4) When waste is separated, college students will consider the level of convenience and economic cost, which will also affect their choice. This study provides a new idea for research on waste separation of specific target college students and provides a reference for future research on related topics in the field of social marketing.

Second, from a practical point of view, suggestions can be put forward regarding the dilemma of waste separation according to the research results.

1. College students with strong behavior and attitudes are more likely to choose waste separation. First, the school can promote the concept of waste separation through the student union, associations, and other channels to promote the formation of the waste separation attitude of college students; innovation in the form and content of publicity is the prerequisite to fully attracting the attention of college students. For example, we can organize class meetings of environmental protection education films and arrange visits to waste separation and recycling education bases to improve students' sensitivity to the environment and pollution perception, to further form a benign atmosphere in the school, and to drive students' value judgment on waste separation to better participation levels in waste separation.
2. When college students are in an atmosphere that tends to encourage involvement in waste separation, their rational motivation for waste separation will be stimulated. When college students live in an environmentally friendly society, they will pay attention to environmental problems and think about how to solve the problem of waste separation. College students tend to believe that most people around them are like-minded and that they should take action to change the environment. Schools can consider how to close the link between the low participation rate of waste separation and the high participation rate of college students. For example, it is possible to set up environmental protection associations, hold contests related to environmental protection, and establish virtual environmental protection communities [5]. However, after the establishment of the virtual account of college students in the virtual community, the issues of how to activate the community, how to enhance the sense of belonging of members, how to make the norms and culture of the virtual community into the real world, and how to cultivate the habit of environmental protection of college students present great challenges. If the virtual community cannot make the best use of its resources, it can only be used as a channel to publicize environmental protection knowledge and appeal for environmental protection, which is no different from the current new media propaganda method advocating waste separation. The proposition of community operation needs to be solved with interdisciplinary theoretical knowledge, such as journalism and communication and marketing. In addition, after the successful establishment of virtual communities, online and offline joint interaction can be conducted to share environmental protection experiences such as waste separation to enhance the experience. At this time, community opinion leaders should also implement their maximum effect, which will improve the intention of college students to participate in waste separation.
3. The difficulty of waste separation and the perception of obstacles to implementation also affect the judgment of waste separation by college students and their confidence in their ability to implement waste separation. Even though college students' views and value judgments on waste separation are positive, they will be restricted by practical factors. Therefore, guidance strategies to improve the existing situation can be put forward from the perspective of improving convenience and reducing economic cost, such as placing recycling facilities in close proximity to users and creating intelligent facilities and easy collection methods. A higher waste separation level and smaller capacity of waste separation facilities will make college students have a reserved attitude toward waste separation. In addition, the cost of waste separation will undoubtedly affect the degree of students' participation in waste separation. According to the rational hypothesis, the economic rewards of waste separation will encourage the enthusiasm of college students. Schools can establish waste separation as a social practice project, and college students who complete relevant indicators can be given credits. On the other hand, college students should be encouraged to believe that they can engage in waste separation, which will make them determined to change their existing habits and improve their self-efficacy, which will in turn create the behavioral motivation of waste separation.
4. Cultivation is environmentally friendly and benefits waste separation habits. Even if college students have a strong attitude toward environmental protection, people around them actively participate in waste separation, and it is easier to carry out waste separation, and they can still reduce their frequency of waste separation because of strong and deep-rooted “bad habits.” At this time, emphasizing the enhancement of environmental protection publicity and the education effect is minimal and lacks practical significance. Therefore, schools and relevant departments should not neglect the problem and practical operation of how to cultivate good waste separation habits of college students. This question is more practical than theoretical propaganda but also more challenging. Schools can cultivate the waste separation habits of college students in virtual environmental protection communities and extend online behavior patterns to offline ones.
5. Habits take time to accumulate, but individuals are eventually able to perform certain behaviors in certain situations consciously and without much thought. The development of a habit is a long and complex process, whether it is developing a new habit or changing a “bad habit” to a good habit. New studies focusing on the field of habits, such as dividing the dimensions of habits and examining the habit scale, can enable schools and relevant departments to put forward more targeted and action-oriented suggestions on improving the participation rate of college students in waste separation behavior.

### 6.4. Future Search

Although this study constructs a model of the waste separation behavior of college students on the basis of planned behavior theory, puts forward relevant conclusions and suggestions, and strives to be scientific in its research, due to the lack of ability and limited experimental and research conditions, there is some potential for future work.

First, the questionnaire method adopts the self-report method, which makes the collected data have some deviation. A small number of 400 valid questionnaires were collected. In addition, there were more females and fewer males among the respondents; thus, it cannot be excluded that the research results may differ due to gender bias. Therefore, the sample of this study cannot fully reflect the general situation of waste separation behavior of college students in Guangzhou Higher Education Mega Center.

Second, in terms of measurement, the SRHI habit scale used in this study has not been widely verified by scholars, and the measurement method still needs to be studied. Other variables can be studied in the future to improve the waste separation behavior model of college students and provide more theoretical support for the waste separation behavior of college students.

Third, in terms of variable extraction, this study only uses one dimension for multiple variables, without considering the dimension division of these variables. In addition, the variables studied in this study are limited, and a complete and comprehensive waste separation model for college students cannot be established. In future studies, the implicit attitudes of respondents need to be explored. In addition, to keep the attention of domestic and foreign scholars in the field of habit research, in the future, adopting an effective method of updating constantly, improving the accuracy of measuring habits, and proposing feasible suggestions from the habit aspect can improve the environmental behavior of college students.

## Figures and Tables

**Figure 1:** Influence mechanism model of waste separation behavior of undergraduate students.

**Table 1:** Measurement of the variables.

Variable	Measuring item	Reference source
Behavioral attitude	A1. It makes sense for me to waste separation	Ghani et al. [59]
	A2. It is necessary for me to waste separation	
	A3. It is pleasant for me to waste separation	

Subjective norm	SN1. The extent to which my family has influenced my waste separation	Mak et al. [39]
	SN2. The extent to which my friends influence my waste separation	
	SN3. The degree of influence of public opinion media on my waste separation	

Perceived behavioral control	PBC1. I can waste separation very easily	Fan et al. [50]
	PBC2. Waste separation behavior is entirely up to me, not objective reasons	
	PBC3. As long as I am willing, I believe I can do waste separation	
Environmental awareness	HH1. I am constantly aware of whether my actions or those of others are beneficial to environmental protection	
	HH2. I often remind myself to form a low-carbon and environmentally friendly lifestyle	

Habit	H1. It's not always possible for me to do waste separation	Glick et al. [31]
	H2. As far as I am concerned, waste is not classified	
	H3. So far, I have not been able to insist on waste separation	
	H4. You do not realize you've separated your trash until you've taken it out	
	H5. You do not realize you've separated your trash until you've taken it out	
	H6. I need to work hard to do waste separation	
	H7. It is very difficult for me to waste separation	
	H8. It would be strange if we deliberately separated the waste one day	
	H9. I need to consider whether I should separate the rubbish	

Intention	BI1. I'm going to stick to waste separation	Chan et al. [48]
	BI2. I was able to separate out the waste as planned	

Behavior	B1. I mixed all the household waste I produced	Masud et al. [33]
	B2. I separate the rubbish into plastic bottles/paper and cartons/kitchen waste/others	

Convenience	RC1. The accessibility of waste separation points will affect my separating behavior	Bagozzi et al. [38]
	RC2. The waste collection point is very close to where I live	
	RC3. If I could set up professional waste separation and recycling facilities, I would be more willing to carry out waste separation	

Economic cost	DD1. I would like to do more expensive but environmentally friendly waste separation	Lu et al. [28]
	DD2. I can accept the requirement that there is a fee for waste separation	
	DD3. If the waste separation behavior can get economic returns, my behavior intention will be stronger	

Personal responsibility	RES1. Everyone is responsible for protecting the environment in his daily life	Setiawan et al. [49]
	RES2. In order to protect the environment, every consumer has the responsibility to separate their waste	

**Table 2:** Sample structure of pretest.

Table of sample characteristics	Project	Additional copies	Percentage (%)
Gender	Male	56	37.6
	Female	93	62.4

Education	College	19	12.8
	University degree	100	67.1
	Postgraduate	30	20.1

Types of colleges and universities	Comprehensive	94	63.1
	Institute of class	21	14.1
	Agriculture, forestry, and class	5	3.3
	Normal class	12	8.1
	Finance and economics	14	9.4
	Other	3	2.0

Professional types	Science and engineering	51	34.2
	One liberal art	98	65.8

Average monthly income	Less than 1000 yuan	24	16.1
	1000–2000 yuan	104	69.8
	2000–3000 yuan	17	11.4
	More than 3000 yuan	4	2.7

**Table 3:** Reliability analysis of each variable in the pretest.

Measured variable	Cronbach's alpha	Item number
Behavior attitude	0.759	3
Subjective norms	0.748	3
Perceptual behavioral control	0.710	3
Intention	0.768	9
Habit	0.856	2
Convenience	0.597	3
Economic costs	0.588	3
Environmental awareness	0.730	2
Personal responsibility	0.828	2
Behavior	0.761	2

**Table 4:** Result of KMO and Bartlett's test in pretest.

KMO sampling suitability quantity		0.618
Bartlett's sphericity test	Approximate chi-square	2108.520
	Degrees of freedom	496
	Significant	0.000

**Table 5:** Description statistics.

Table of sample characteristics	Project	Additional copies	Percentage (%)
Gender	Male	158	39.5
	Female	242	60.5

Education	College	52	13.0
	University degree	204	51.0
	Postgraduate	144	36.0

Types of colleges and universities	Comprehensive	268	67.0
	Institute of class	45	11.2
	Agriculture, forestry, and class	11	2.8
	Normal class	31	7.7
	Finance and economics	40	10.0
	Other	5	1.3

Professional types	Science and engineering	103	25.8
	One liberal art	297	74.2

Average monthly income	Less than 1000 yuan	51	12.7
	1000–2000 yuan	308	77.0
	2000–3000 yuan	34	8.5
	More than 3000 yuan	7	1.8

**Table 6:** Reliability analysis.

Measured variables	Cronbach's alpha	Item number
Behavior attitude	0.811	3
Subjective norms	0.805	3
Perceptual behavioral control	0.739	3
Intention	0.880	9
Habit	0.899	2
Convenience	0.983	2
Economic costs	0.788	2
Environmental awareness	0.713	2
Personal responsibility	0.824	2
Behavior	0.783	2

**Table 7:** Result of KMO and Bartlett's test.

KMO Kaiser–Meyer–Olkin measure of sampling adequacy		0.779
Bartlett's sphericity test	The approximate chi-square	5799.182
	Variance	435
	Significant	0.000

**Table 8:** Correlation analysis.

	Behavior attitude	Subjective norms	Perceptual behavioral control	Intention	Habit	Convenience	Economic costs	Environmental awareness	Personal responsibility	Behavior
Behavior attitude	1									
Subjective norms	0.193^*∗∗*^	1								
Perceptual behavioral control	0.262^*∗∗*^	0.262^*∗∗*^	1							
Intention	0.247^*∗∗*^	0.235^*∗∗*^	0.239^*∗∗*^	1						
Habit	0.197^*∗∗*^	0.205^*∗∗*^	0.181^*∗∗*^	0.188^*∗∗*^	1					
Convenience	0.202^*∗∗*^	0.217^*∗∗*^	0.191^*∗∗*^	0.188^*∗∗*^	0.171^*∗∗*^	1				
Economic costs	−0.236^*∗∗*^	−0.177^*∗*^	−0.265^*∗∗*^	−0.223^*∗∗*^	−0.191^*∗∗*^	−.223^*∗∗*^	1			
Environmental awareness	0.251^*∗∗*^	0.200^*∗∗*^	0.257^*∗∗*^	0.215^*∗∗*^	0.182^*∗∗*^	0.187^*∗∗*^	−0.377^*∗∗*^	1		
Personal responsibility	0.258^*∗∗*^	0.206^*∗∗*^	0.194^*∗∗*^	0.227^*∗∗*^	0.208^*∗∗*^	0.233^*∗∗*^	−0.243^*∗∗*^	0.299^*∗∗*^	1	
Behavior	0.196^*∗∗*^	0.190^*∗∗*^	0.187^*∗∗*^	0.316^*∗∗*^	0.204^*∗∗*^	0.191^*∗∗*^	−0.186^*∗∗*^	0.204^*∗∗*^	0.182^*∗∗*^	1
Average	4.066	3.507	3.580	3.556	2.816	4.022	2.598	3.645	3.989	3.102
Standard deviation	0.630	0.857	0.708	0.834	0.790	0.823	0.843	0.856	0.886	1.075

*Note*. ^*∗*^At 0.05 level (two-tailed), the correlation was significant. ^*∗∗*^At 0.01 level (two-tailed), the correlation was significant. ^*∗∗∗*^At 0.001 level (two-tailed), the correlation was significant.

**Table 9:** Rotated component matrix^a^.

	Element									
	1	2	3	4	5	6	7	8	9	10
Habit 1	0.727	−0.088	−0.051	0.011	0.010	0.040	−0.006	0.032	−0.142	0.011
Habit 7	0.726	0.023	−0.013	0.019	−0.053	0.051	−0.088	−0.023	−0.070	0.039
Habit 9	0.716	−0.067	0.058	−0.019	0.061	0.010	−0.034	0.073	−0.034	0.022
Habit 5	0.716	−0.064	0.091	−0.126	−0.030	0.022	0.020	0.013	0.011	0.151
Habit 3	0.714	0.033	0.013	0.061	−0.033	−0.111	0.014	0.012	−0.003	−0.183
Habit 2	0.709	0.020	−0.049	0.035	−0.005	−0.183	−0.114	−0.020	−0.114	−0.057
Habit 4	0.703	−0.002	−0.035	0.025	0.009	0.112	0.046	0.039	0.033	−0.092
Habit 6	0.701	−0.102	0.015	−0.099	−0.029	−0.048	−0.025	−0.032	0.017	0.049
Habit 8	0.701	0.000	0.026	−0.035	0.013	−0.117	0.000	0.044	−0.036	−0.115
Behavior attitude 1	−0.118	0.872	0.144	0.114	0.050	0.066	0.118	−0.060	0.055	0.058
Behavior attitude 2	−0.064	0.859	0.158	0.050	0.051	0.069	0.170	−0.130	0.053	0.043
Behavior attitude 3	−0.018	0.728	−0.100	0.094	0.073	0.085	−0.049	−0.012	0.050	0.118
Subjective norm 2	0.033	0.030	0.885	0.031	0.093	0.038	0.097	−0.025	0.028	0.039
Subjective norm 1	0.033	0.017	0.869	0.040	0.007	0.048	0.034	−0.080	0.074	0.028
Subjective norm 3	−0.007	0.125	0.712	0.246	0.104	0.128	0.037	−0.026	0.061	0.091
Perceptual behavioral control 2	−0.022	0.068	0.096	0.833	−0.006	0.025	0.042	−0.026	0.111	0.053
Perceptual behavioral control 1	−0.019	−0.019	0.106	0.788	0.008	0.178	0.003	−0.098	0.011	0.141
Perceptual behavioral control 3	−0.046	0.254	0.077	0.711	0.176	−0.004	0.115	−0.110	0.019	0.025
Convenience 2	−0.009	0.088	0.093	0.073	0.964	0.059	0.084	−0.090	0.065	0.078
Convenience 1	−0.017	0.090	0.105	0.077	0.961	0.073	0.099	−0.077	0.080	0.046
Intention 2	−0.079	0.085	0.102	0.105	0.047	0.906	0.053	−0.091	0.142	0.053
Intention 1	−0.051	0.143	0.109	0.098	0.088	0.900	0.113	−0.065	0.121	0.070
Personal responsibility 1	−0.073	0.079	0.065	0.109	0.098	0.025	0.886	−0.072	0.078	0.132
Personal responsibility 2	−0.052	0.122	0.098	0.035	0.080	0.134	0.878	−0.092	0.034	0.092
Economic cost 2	0.049	−0.073	−0.105	−0.126	−0.086	−0.053	−0.058	0.883	−0.079	−0.091
Economic cost 1	0.051	−0.114	−0.026	−0.094	−0.079	−0.100	−0.113	0.849	−0.035	−0.220
Behavior 1	−0.097	0.102	0.112	0.060	0.085	0.112	0.064	−0.060	0.868	0.047
Behavior 2	−0.145	0.045	0.045	0.081	0.054	0.135	0.045	−0.051	0.867	0.086
Environmental awareness 2	−0.043	0.123	0.088	0.096	0.038	0.023	0.174	−0.128	0.041	0.824
Environmental awareness 1	−0.065	0.100	0.061	0.123	0.083	0.094	0.055	−0.171	0.096	0.820

**Table 10:** Regression analysis of economic cost and convenience on perceived behavior control.

Variable		Dependent variable-behavior-perceived behavioral control	
		Model 2.1	Model 2.2
Control variables	Gender	0.004	−0.002
	Education background	−0.060	−0.057
	Institution type	0.068	0.066
	Professional types	0.071	0.080
	Average monthly income	0.007	0.001

Independent variable	Economic cost	−0.257^*∗∗∗*^	
	Convenience		0.182^*∗∗∗*^
	Adjusted *R*^2^	0.069	0.036
	Variation in *R*^2^	0.065^*∗∗∗*^	0.032^*∗∗∗*^
	F value	5.954^*∗∗∗*^	3.480^*∗∗*^

**Table 11:** Analysis of the mediating effect of behavioral intention on behavioral attitude-waste separation behavior.

Variable		Dependent variable-behavior		
		Model 3.1	Model 3.2	Model 3.3
Control variables	Gender	0.047	0.132^*∗∗*^	0.008
	Education background	−0.001	−0.116^*∗*^	0.033
	Institution type	0.035	0.044	0.022
	Professional types	0.135^*∗∗*^	−0.037	0.146^*∗∗*^
	Average monthly income	−0.005	−0.041	0.007

Independent variable	Behavior attitude	0.183^*∗∗∗*^	0.228^*∗∗∗*^	0.117^*∗*^
	Behavioral intention			0.290^*∗∗∗*^
	Adjusted *R*^2^	0.048	0.083	0.123
	Variation in *R*^2^	0.032^*∗∗∗*^	0.050^*∗∗∗*^	0.108^*∗∗∗*^
	F value	4.338^*∗∗∗*^	7.007^*∗∗∗*^	8.991^*∗∗∗*^

**Table 12:** Regression analysis of environmental awareness and personal responsibility on behavior and attitude.

Variable		Dependent variable-behavior attitude	
		Model 1.1	Model 1.2
Control variables	Gender	−0.06	−0.010
	Education background	−0.114^*∗*^	−0.125^*∗*^
	Institution type	−0.042	−0.029
	Professional types	0.094	0.075
	Average monthly income	−0.083	−0.075

Independent variable	Environmental awareness	0.235^*∗∗∗*^	
	Individual accountability		0.237^*∗∗∗*^
	Adjusted *R*^2^	0.080	0.081
	Variation in *R*^2^	0.054^*∗∗∗*^	0.055^*∗∗∗*^

**Table 13:** Analysis of the mediating effect of behavioral intention on subjective norms-waste separation behavior.

Variable		Dependent variable-behavior		
		Model 3.1	Model 3.2	Model 3.3
Control variables	Gender	0.031	0.112^*∗*^	−0.002
	Education background	−0.009	−0.126^*∗*^	0.028
	Institution type	0.025	0.033	0.016
	Professional types	0.136^*∗∗*^	−0.036	0.147^*∗∗*^
	Average monthly income	−0.024	−0.063	−0.005

Independent variable	Subjective norms	0.170^*∗∗*^	0.213^*∗∗∗*^	0.107^*∗*^
	Behavioral intention			0.294^*∗∗∗*^
	Adjusted *R*^2^	0.043	0.076	0.121
	Variation in *R*^2^	0.028^*∗∗*^	0.044^*∗∗∗*^	0.107^*∗∗∗*^
	*F* value	4.016^*∗∗*^	6.501^*∗∗∗*^	8.855^*∗∗∗*^

**Table 14:** Analysis of the mediating effect of behavioral intention on perceived behavioral control-waste separation behavior.

Variable		Dependent variable-behavior		
		Model 3.1	Model 3.2	Model 3.3
Control variables	Gender	0.044	0.129^*∗∗*^	0.006
	Education background	−0.016	−0.134^*∗∗*^	0.023
	Institution type	0.018	0.022	0.011
	Professional types	0.137^*∗∗*^	−0.037	0.148^*∗∗*^
	Average monthly income	−0.020	−0.059	−0.003

Independent variable	Perceptual behavioral control	0.170^*∗∗*^	0.228^*∗∗∗*^	0.104^*∗*^
	Behavioral intention			0.293^*∗∗∗*^
	Adjusted *R*^2^	0.044	0.084	0.120
	Variation in *R*^2^	0.029^*∗∗*^	0.051^*∗∗∗*^	0.106^*∗∗∗*^
	*F* value	4.063^*∗∗*^	7.089^*∗∗∗*^	8.807^*∗∗∗*^

**Table 15:** Analysis of moderating effects.

Variable		Dependent variable-behavior			
		Model 4.1	Model 4.2	Model 4.3	Model 4.4
Control variables	Gender	0.047	0.005	−0.001	−0.009
	Education background	−0.027	0.020	0.035	0.039
	Institution type	0.029	0.017	0.023	0.020
	Professional types	0.153^*∗∗*^	0.158^*∗∗*^	0.169^*∗∗∗*^	0.175^*∗∗∗*^
	Average monthly income	−0.021	−0.002	−0.005	−0.010

Independent variable	Behavioral intention		0.317^*∗∗∗*^	0.289^*∗∗∗*^	0.273^*∗∗∗*^
	Habit			0.166^*∗∗*^	0.156^*∗∗*^
	Behavioral intention × habit				−0.099^*∗*^
	Adjusted *R*^2^	0.018	0.113	0.137	0.144
	Variation in *R*^2^	0.030^*∗*^	0.96^*∗∗∗*^	0.026^*∗∗*^	0.009^*∗*^
	*F* value	2.426^*∗*^	9.435^*∗∗∗*^	10.034^*∗∗∗*^	9.387^*∗∗∗*^

**Table 16:** Summary of hypothesis verification results.

Serial number	Hypothesis	Result
H1	College students' attitude toward waste separation behavior has a significant positive impact on waste separation behavior	Valid
H2	The subjective norms of waste separation behavior of college students have a significant positive influence on waste separation behavior	Valid
H3	The perceptual behavior control of college students has a significant positive influence on waste separation behavior	Valid
H4	The behavioral intention of waste separation plays a mediating role between attitude and waste separation behavior	Valid
H5	The behavioral intention of waste separation plays an intermediary role between the subjective norm and waste separation behavior	Valid
H6	The behavioral intention of waste separation plays a mediating role between perceived behavioral control and waste separation behavior	Valid
H7	The behavior habit of waste separation plays a moderating role between the behavioral intention and waste separation behavior of college students	Valid
H8	The environmental awareness of college students has a significant positive influence on their attitude	Valid
H9	College students' personal responsibility has a significant positive influence on their attitude	Valid
H10	The convenience of waste separation behavior has a significant positive influence on the perceived behavior control of college students	Valid
H11	The economic cost of waste separation has a significant negative influence on perceived behavior control of college students	Valid

## Data Availability

The data used to support the findings of this study are included within the article.
